# Improvement of Bronchial Immune Hypersensitivity Reaction Using Extracts from *Chrysanthemum morifolium* Ramatuelle and *Scutellaria baicalensis* Georgi

**DOI:** 10.1155/2021/3173823

**Published:** 2021-12-11

**Authors:** Kyoungwon Cho, Sung Sun Park, Hakjoo Choi

**Affiliations:** ^1^R&D Division, Chong Kun Dang Healthcare Corporation, Seoul 07249, Republic of Korea; ^2^R&D Center, CH Labs Corporation, Seoul 07249, Republic of Korea; ^3^College of Pharmacy, Chungnam National University, Daejeon 34134, Republic of Korea; ^4^Department of Herbology, College of Oriental Medicine, Dae-Gu Haany University, Daegu 42158, Republic of Korea

## Abstract

*Chrysanthemum morifolium* Ramatuelle and *Scutellaria baicalensis* Georgi (skullcap) have been used as safe raw materials for drinking or as traditional medicines in Korea. In this study, we investigated the potential therapeutic effects of ovalbumin-induced asthma in a mouse model. After establishing the model, mice were treated with a mixture of chrysanthemum and skullcap extracts at different mixing ratios (6 : 4, 7 : 3, and 8 : 2). Immune cell counts and the production of various inflammatory cytokines were measured using biochemical tests. Among the mixtures tested, the 7 : 3 ratio (CS73) showed the most pronounced effects. CS73 significantly reduced the levels of the inflammatory cytokines interleukin- (IL-) 1*β*, IL-4, IL-5, IL-6, IL-10, IL-13, IL-17A, IL-17F, and IL-17E in the serum and bronchoalveolar lavage fluid of asthmatic mice. In addition, CS73 treatment significantly increased the production of IL-2 and interferon-*γ* and decreased the production of immunoglobulin E, histamine, and thymic stromal lymphopoietin in asthmatic mice compared to the control group. Our results suggest that the combination of chrysanthemum and skullcap extracts, especially at a 7 : 3 ratio, can be used to improve bronchial health and contribute to improved public health.

## 1. Introduction

Although recent advances in molecular biology and medicine have led to the development of various treatment methods for allergic diseases, including asthma, the number of cases of allergic disease continues to increase because of complex pathology and environmental changes [1]. Environmental factors that cause a rapid increase in the number of patients with allergies include a westernized diet, atmospheric pollution by chemical fuels, fewer bacterial or parasitic infections, and increased psychological stress [2]. Medicines currently used to treat asthma include chemical mediator release inhibitors, antihistamines, and Th2 cytokine production inhibitors. In addition, steroids, anticholinergics, and *α-* and *β*_2_-receptor agonists in various forms, including topical drugs and inhalers, are used. However, these treatments cannot completely treat the root causes of asthma [3]. As atmospheric pollution in Korea continues to increase because of the presence of fine particulate matter and yellow dust, we aimed to identify functional materials derived from natural substances that can alleviate bronchial discomfort by improving bronchial hyperresponsiveness.

Among the natural resources that are native to Korea, chrysanthemum (*Chrysanthemum morifolium* Ramatuelle) and skullcap (*Scutellaria baicalensis* Georgi) are safe raw materials that have long been consumed as a tea or used as herbal medicines [4]. Previous studies have shown that chrysanthemum and skullcap can alleviate acute lung injury [5, 6]. Furthermore, an *in vitro* study showed that compared to a single treatment with chrysanthemum or skullcap extracts, a mixture of both extracts was more effective in relieving inflammatory responses in PMA-treated A549 and NCI-H292 cells [7]. However, the effects of the mixture have not been clarified in animal studies. This study aimed to investigate the therapeutic potential of a mixture of chrysanthemum and skullcap extracts in ovalbumin- (OVA-) treated mice.

## 2. Materials and Methods

### 2.1. Samples

Chrysanthemum flowers and the roots of the skullcap used were purchased from the Korea Medicine Herbal Association and Gyeongdong Market (Seoul, Korea). Plants were identified by the Korea Medicine Herbal Association, which is under the jurisdiction of the Ministry of Agriculture, Food, and Rural Affairs. Chrysanthemum flowers (90 kg) were extracted using 70% ethanol at 75°C for 12 h and subsequently concentrated. After maltodextrin was added, the extract was spray-dried. The yield from the chrysanthemum was 34.78%. Ninety kilograms of skullcap roots were extracted using hydrothermal extraction at 95°C. After maltodextrin was mixed, the extract was spray-dried. The final extraction yield was 89%.

### 2.2. High-Performance Liquid Chromatography (HPLC) Analysis

For HPLC analysis of chrysanthemum and skullcap extracts and their active compounds luteolin 7-glucoside [8] and baicalein [9], respectively, we used the analytical HPLC system (Waters e2695; Waters Co., Milford, MA, USA) equipped with a Waters XSelect HSS C_18_ column (4.6 mm × 250 mm, 5 *μ*m) at 40°C with a flow rate of 1.0 mL/min. For the detection of compounds in each extract, we used a photodiode array detector (2998 PDA Detector; Waters Co., Milford, MA, USA). For chrysanthemum extract and luteolin 7-glucoside (Sigma-Aldrich, St. Louis, MO, USA) analysis, the mobile phase contained 0.1% trifluoroacetic acid in water (phase A) and acetonitrile (ACN) (phase B). The HPLC run was programmed as follows: 0–25 min, 15%–40% phase B; 25–26 min, 40%–100% phase B; 26–30 min, 100% phase B; 30–31 min, 100%–15% phase B; and 31–35 min, 15% phase B. The detection wavelength was set to 330 nm. For the skullcap extract and baicalein (Sigma-Aldrich, St. Louis, MO, USA) analysis, 1% acetic acid in water (phase A) and 1% acetic acid in ACN (phase B) were used and the HPLC run was programmed as follows: 0–10 min, 25%–32% phase B; 10–20 min, 32%–45% phase B; 20–24 min, 45% phase B; and 24–35 min, 45%–48% phase B. The detection wavelength was set to 277 nm. The peaks of luteolin 7-glucoside and baicalein from the extracts were identified by comparison with the retention times of the standards, and the UV spectra were also compared between compounds and extracts.

### 2.3. Experimental Animals and Animal Care

Eighty-eight five-week-old male BALB/c mice (20–22 g) were provided by Samtako Co. Ltd. (Osan, Korea). The mice had *ad libitum* access to standard rodent chow and water until the day of the experiment. The mice were housed in a controlled environment under a 12 h light/dark cycle at 22 ± 2°C and humidity of 55% ± 15% for a 2-week adaptation period before the experiment. Mice were classified into 11 groups (*n* = 8 per group): negative control group with no treatment, control group with asthma induction and oral administration of distilled water, experimental groups with oral administration of 50, 100, or 200 mg/kg body weight (BW) of chrysanthemum and skullcap sample mixed in a 6 : 4, 7 : 3 (CS73), or 8 : 2 ratio. For the animal experiments, when chrysanthemum and skullcap were tested at a concentration of 320–1280 mg/kg BW and 800–5000 mg/kg BW, respectively, neither of them showed immune cell-related toxicity in hematological data [10, 11]. Based on the results of these studies, the experiment was performed at a lower concentration. All experiments were approved by the Daejeon University Institutional Animal Care and Use Committee (approval no. DJUARB2017-018).

### 2.4. Mouse Model of OVA-Induced Asthma and Treatments

To establish an animal model of OVA-induced asthma, mice were intraperitoneally administered 0.3 mL of 1 : 1 1 mg OVA (chicken egg albumin) in phosphate-buffered saline (PBS): aluminum hydroxide gel once every 7 days. From day 21 onwards, i.e., 7 days after the last intraperitoneal injection, mice were placed in 50 × 15 × 50 cm acrylic boxes and exposed to 50 mL of aerosolized OVA solution (2 mg/mL) for 30 min once every other day (on days 21, 23, 25, 27, and 29) for asthma induction. Aerosolized OVA was generated using a nebulizer. The experiments were conducted for 2 weeks after the intraperitoneal injections were administered.

### 2.5. Measurement of Immune Cells in the Blood and Bronchoalveolar Lavage Fluid (BALF)

At the end of the experiment, whole blood was collected via cardiac puncture and analyzed at KPNT (Cheongju, Korea) for white blood cell and eosinophil counts.

### 2.6. Cell Isolation from the Lungs and Bronchial BALF

At the end of the experiment, the lungs of the mice were dissected. For cell isolation from BALF, a 24G catheter was inserted into the trachea and secured with a suture thread. A syringe containing Dulbecco's Modified Eagle's medium (DMEM) was attached to the catheter, and three pulsatile aspirations were performed to obtain BALF. Next, 100 *μ*L of ammonium-chloride-potassium buffer was added to the collected BALF, and the sample was incubated for 5 min at 37°C to lyse the red blood cells. The sample was subsequently washed with culture medium and stained with 0.04% trypan blue to determine the immune cell count.

### 2.7. Separation of Serum and BALF Supernatant

At the end of the experiment, blood samples were collected via cardiac puncture under anesthesia using ethyl ether and centrifuged at 3000 rpm for 15 min to separate the serum. The separated BALF cells were adjusted to a density of 5 × 10^5^ cells and incubated in Dulbecco's modified Eagle medium containing 10% fetal bovine serum at 37°C in a 5% CO_2_ atmosphere for 24 h. Next, the mixture was centrifuged at 1200 rpm for 5 min to separate the culture medium, and the supernatant was aspirated.

### 2.8. Measurement of Cytokine Production in Serum and BALF

Serum and supernatant (25 *μ*L) isolated from the mice along with cytokine standards were added to each well of a 96-well plate, followed by the addition of 25 *μ*L of matrix buffer, 25 *μ*L of assay buffer, and 25 *μ*L of antibody-immobilized beads. The plate was incubated for 2 h at 25°C and subsequently washed twice with washing buffer. Next, 25 *μ*L of the detection antibody was added, and the plate was incubated for 1 h at 25°C, followed by the addition of 25 *μ*L of streptavidin-phycoerythrin and incubation for 30 min at 25°C. The plate was washed twice with a washing buffer solution. PBS (150 *μ*L) was added, and the plate was placed on a shaker for 5 min and Fluorescence emitted from beads was measured using a Luminex 200 system (Luminex, Austin, TX, USA).

### 2.9. Measurement of OVA-Specific Immunoglobulin (Ig)E Production in Serum and BALF

Serum and its supernatant (50 *μ*L) isolated from mice and the IgE standard were added to each well of a 96-well ELISA plate, followed by the addition of matrix buffer (50 *μ*L) and assay buffer (50 *μ*L). The plate was incubated for 2 h at 25°C and was subsequently washed four times with washing buffer. Next, 100 *μ*L of the detection antibody was added to each well, followed by incubation for 1 h at 25°C. The plate was further washed four times with washing buffer. Avidin-HRP (100 *μ*L) was added, and the mixture was incubated for 30 min at 25°C. Finally, the plate was washed four times with washing buffer, followed by the addition of a substrate solution (100 *μ*L). The plates were incubated in the dark for 15 min at 25°C. Stop solution (100 *μ*L) was added, and the absorbance was measured at 450 nm.

### 2.10. Measurement of Histamine Production Level in Plasma and BALF

One hundred microliters of separated serum, supernatant, and histamine standards were dispensed into each well of a 96-well ELISA plate. Next, 10 *μ*L of balance solution and 50 *μ*L of the conjugate were added and incubated at 37°C for 1 h. After washing five times with a washing buffer, 50 *μ*L of each of substrates A and B was added and reacted at 37°C for 15 min. Subsequently, 50 *μ*L of the stop solution was added, and the optical density was measured at 450 nm.

### 2.11. Measurement of Thymic Stromal Lymphopoietin (TSLP) Level in Plasma and BALF

Fifty microliters of the separated serum, supernatant, and TSLP standard were dispensed into each well of a 96-well ELISA plate. Next, 50 *μ*L of the RD1-21 reagent was added, mixed, and reacted at room temperature for 2 h. After washing five times with washing buffer, 100 *μ*L of TSLP conjugate was added and incubated at room temperature for 2 h. The wells were washed five times, and 100 *μ*L of the substrate solution was added and incubated in the dark at room temperature for 30 min. Finally, 100 *μ*L of stop solution was added, and the absorbance was measured at 450 nm.

### 2.12. Statistical Analysis

Data are expressed as mean ± standard deviation (SD) of eight mice in each group. Statistical analysis of the experimental data was performed using the unpaired Student's *t*-test and ANOVA using SPSS version 18.0 (IBM, Armonk, NY, USA). Three significance levels were considered: ^*∗*^*p* < 0.05, ^*∗∗*^*p* < 0.01, and ^*∗∗∗*^*p* < 0.001.

## 3. Results and Discussion

### 3.1. HPLC Chromatogram

There are various compounds in chrysanthemum and skullcap, among which there is data that chrysanthemum contains luteolin 7-glucoside [8] and skullcap contains baicalin [9]. Luteolin 7-glucoside and baicalein have protective effects against respiratory diseases such as asthma, ischemia, and reperfusion-induced lung injury [12, 13]. Accordingly, the presence of the active compounds luteolin 7-glucoside and baicalein in the chrysanthemum and skullcap extracts was confirmed using HPLC. The results of the HPLC analysis of the extracts and their active compounds are shown in Figure 1. The peak of the standard luteolin 7-glucoside was detected at 8.797 min, which was also detected at 9.101 min among the peaks of the chrysanthemum extract. The peak of the standard baicalein was detected at 17.559 min, which was also detected at 17.461 min among the peaks of the skullcap extract. In addition, the UV spectra of luteolin 7-glucoside and luteolin 7-glucoside in chrysanthemum extracts were identical. Likewise, the pattern of the UV spectrum of baicalein itself and baicalein in the skullcap extract was the same (Figure 1).

After mixing the chrysanthemum and skullcap extracts according to the ratios of 6 : 4, 7 : 3, and 8 : 2, we analyzed HPLC chromatograms and UV spectrum. As shown in Figure 2, HPLC chromatograms patterns were similar. In particular, luteolin 7-glucoside in mixtures of chrysanthemum and skullcap extracts was detected at 9.054 min in a 6 : 4 ratio, 9.101 min in 7 : 3 ratio, and 9.109 min in 8 : 2 ratio, and baicalein was also identified at 17.486 min in 6 : 4 ratio, 17.461 min in 7 : 3 ratio, and 17.460 min in 8 : 2 ratio. The UV spectrum pattern of each compound in each mixture was similar to that in Figure 1.

### 3.2. Effects of Chrysanthemum and Skullcap Mixtures on Immune Factors

In a previous study, we conducted an *in vitro* experiment on the effects of single and combined treatments of chrysanthemum and skullcap extracts on NCI-H292 cells [7]. The study results showed that combined treatment with ratios of 8 : 2 and 6 : 4 was more effective than treatment with chrysanthemum and skullcap alone. Therefore, in this study, mixtures of chrysanthemum and skullcap extract at ratios of 8 : 2, 7 : 3, and 6 : 4 were tested. The 7 : 3 ratio showed the highest effect on different parameters compared to the other groups (Table 1). Several studies have reported that bronchial-related diseases are alleviated by regulating the expression of immune-related factors, such as a decrease in the levels of IL-1*β* and IL-4 or an increase in IFN-*γ* [14]. In addition, studies have shown that this mechanism is controlled by extracts derived from natural products to protect bronchial tubes [15]. Therefore, these results confirm the value of the extract mixture as a composite that can improve bronchial health and contribute to the health of people affected by fine dust. Furthermore, our findings provide a basis for the potential development of a mixture of chrysanthemum and skullcap extracts as a natural therapeutic formulation to treat asthma.

### 3.3. Effects of CS73 on White Blood Cell (WBC) and Eosinophil Counts

WBCs are related to the immune system and are categorized as granulocytes and agranulocytes [16]. Granulocytes include eosinophils, neutrophils, and basophils, whereas agranulocytes include lymphocytes and monocytes. Some WBCs remove allergens that enter the body via phagocytosis or the generation of antibodies that fight infection [17]. In the present study, WBC counts showed a significant decrease in BALF from the CS73 group compared to the control group (*p* < 0.01). In the CS73-50 group, there was no difference compared with the control group; however, when CS73 was administered at 100 and 200 mg/kg/day, the WBC levels in BALF were significantly decreased. Eosinophils are produced and differentiated by interleukin- (IL-) 5 and contain inflammatory proteins, including major basic proteins, eosinophil-derived neurotoxins, cationic proteins, and peroxidase. Major basic proteins play an important role in the development of asthma as they directly affect bronchial epithelial cells, increase airway hyperresponsiveness, and induce mast cell degranulation. Furthermore, they contain leukotrienes and can increase bronchoconstriction and vascular permeability [18]. Analysis of the eosinophil count showed a significant decrease in the CS73 group compared to that in the control group (*p* < 0.01) (Figure 3).

### 3.4. Effect of CS73 on Th2 Cytokine Production

In the CS73-50 group, there was no difference in WBC levels compared with the control group; however, when CS73 was administered at 100 and 200 mg/kg/day, the WBC levels in BALF were significantly decreased (Figure 4). Th2 cells play an important role in type 2 immune response to ectoparasite and bacterial infections by inducing and developing a humoral immune response via the production of IL-4, IL-5, and IL-13 [19]. IL-1*β* is involved in various cellular activities, including cell proliferation, differentiation, and apoptosis, in response to various stimulants [20]. In a hyperinflammatory state, IL-16 plays an important role as a mediator of the inflammatory response by stimulating the migration of immune cells and increasing the production of cytokines via T cell activation. In addition, IL-16 induces IL-17-mediated asthma [21]. IL-4 plays an important role in promoting the production of IgE, which is a critical factor in the development of asthma. IL-4 also stimulates immune cells and secretes inflammatory mediators, which lead to increased bronchial hyperresponsiveness and airway obstruction [22]. IL-5 is a cytokine that assists in IL-4 production and causes eosinophilia. It activates eosinophils and promotes the secretion of granules from eosinophils, causing an inflammatory response in the airway and bronchial hyperresponsiveness [23]. IL-6 is a cytokine involved in various inflammatory responses, including neutrophil production and regulation of B lymphocyte growth and differentiation [24]. Furthermore, IL-6 contributes to the progression of allergic diseases to the chronic stage and is induced by IL-17 in asthma [25]. IL-10 is an important immunoregulatory cytokine produced by various cell types. It can inhibit inflammatory responses and regulate the proliferation and differentiation of immune cells, including T cells, B cells, NK cells, and antigen-presenting cells [26]. Furthermore, it inhibits the synthesis of proinflammatory cytokines, such as interferon- (IFN-) *γ*, IL-2, IL-3, and GM-CSF, and aggravates asthma. IL-13 induces airway hyperresponsiveness, which is a hallmark of asthma. IL-13 shares receptors with IL-4, as it is functionally similar to IL-4. It also plays an important role in IgE-mediated inflammation and stimulates bronchial epithelial cells or smooth muscle cells, resulting in increased eotaxin secretion and activation of eosinophils, causing an inflammatory response in the airway and bronchial hyperresponsiveness [27].

### 3.5. Effect of CS73 on Th17 Cytokine Production

In this study, the levels of IL-17A, IL-17E, and IL-17F in the serum and BALF were significantly decreased in the CS73 group compared to the control group in a dose-dependent manner (Figure 5). IL-17A is a proinflammatory cytokine produced by activated T cells. It stimulates various immune cell types, including fibroblasts and bronchial smooth muscle cells, to induce several factors and aggravates asthma-induced inflammation and bronchial hyperresponsiveness [28]. IL-17E, also called IL-25, is a cytokine released by bronchial epithelial and immune cells and activates lymphocytes and eosinophils, inducing the production of several cytokines such as IL-4, IL-5, and IL-13 [29]. Therefore, the immune response of Th2 cells is increased, resulting in the development or aggravation of asthma. IL-17F is a proinflammatory cytokine produced by activated T cells. It induces a variety of cytokines, chemokines, and adhesion molecules in bronchial epithelial cells, vein endothelial cells, fibroblasts, and eosinophils, aggravating inflammation and bronchial hyperresponsiveness arising from asthma [21]. Studies have shown that natural extracts relieve asthma by reducing Th17 levels [30].

### 3.6. Effect of CS73 on Th1 Cytokine Production

Th1 cells and macrophages secrete the cytokine IFN-*γ*, which enhances their ability to present antigens to T lymphocytes. Th1 is characterized by the secretion of tumor necrosis factor (TNF), lymphotoxin, and IL-2 [31]. The binding of IL-2 to receptors present on reactive cells promotes T cell proliferation and differentiation, induces B cell proliferation, and activates macrophages. IL-2 is primarily produced via the Th1 cell immune response, plays a role in restoring immune imbalance in asthma, and shows a predominant Th2 cell immune response. Cytokine IFN-*γ* is part of the innate immune system and is involved in immune cell activation and protection of the body against allergens. In addition, Th1 cells are produced to maintain the homeostasis of the Th1/Th2 response [32]. It has been shown that natural extracts such as that from grape seed and propolis relieve asthma by increasing the expression of IL-2 and IFN-*γ* [33, 34]. In this study, the production of IL-2 and IFN-*γ* in the serum and BALF was significantly increased in the CS73 compared to the control group and showed a tendency to increase as the concentration of CS73 increased (Figure 6).

### 3.7. Effects of CS73 on IgE, Histamine, and TSLP Production

Our results showed that IgE, histamine, and TSLP production in the serum and BALF were significantly reduced in the CS73 group compared to those in the control group. Except for TSLP levels in BALF, all parameters were significantly decreased in a dose-dependent manner depending on the sample treatment. Concerning TSLP levels in BALF compared with the control group, significant differences were observed in the CS73_100 and CS72_200 groups, but not with the CS73_50 group (Figure 7). IgE is an immunoglobulin associated with the development of allergic diseases, and it is unbound in the local mucosal tissues and secretions or bound to mast cells [35]. IgE translocates to mast cells or basophils in different parts of the body through the blood. When an allergen enters the body, IgE activates mast cells in the airway and induces the production of several types of inflammatory factors [36]. Therefore, total serum IgE levels were measured and evaluated for the diagnosis of allergic diseases. Histamine is a chemical compound involved in allergic reactions and inflammation. It is released from immune cells, such as macrophages, through antigen-antibody reactions, which leads to the dilation of capillaries, increased permeability (rhinorrhea and edema), bronchoconstriction, and bronchial mucus secretion [37]. TSLP plays an important role in the maturation of T cell groups via activation of antigen-presenting cells and is primarily produced in fibroblasts or epithelial cells [38]. Additionally, antigen-presenting cells are activated by allergens that enter the body from the outside, leading to the maturation of Th2 cells and induction of the Th2 immune response [39].

The main causes of allergic diseases include food allergies, genetic factors, environmental pollution, fine particulate matter, increased antigens from new living environments, and changes in diet [40]. There has been an increase in the number of cases of allergic disease. Recent advances in molecular biology and medicine have enabled in-depth studies on the etiology and pathology of allergies, leading to the identification of various pathological mechanisms. Therefore, new treatment strategies are required based on the mechanisms underlying the development of allergic diseases, and the formulation of novel treatments using herbal medicines made from natural substances has attracted great interest.

Airway hyperresponsiveness refers to the increased sensitivity of the airways to inhaled physical or chemical stimuli and is a characteristic feature of asthma. It is closely associated with airway inflammation. Therefore, increased airway hyperresponsiveness is an important marker of the severity of asthma. In this study, the number of WBCs generated by OVA-induced asthma was decreased in the BALF, whereas eosinophils and basophils were significantly decreased in the CS73 group.

Cytokines are a large group of biologically active substances produced by immune cells and play important roles in the regulation of immunity and defense of the body [41]. Cytokines are associated with the development of allergic inflammation, such as Th2 cell differentiation, IgE production, and eosinophil proliferation [42]. In mice, CD4 T cells are classified as Th1 or Th2 cells, depending on the type of cytokine produced. Th1 cells produce IFN-*γ* and IL-2, and Th2 cells produce IL-4, IL-5, and IL-10, whereas GM-CSF and TNF-*α* are produced by Th1 and Th2 cells. In addition, it is known that differentiation into Th1 cells from precursor cell Th0 is promoted by IL-2, IL-12, and IFN-*γ*, whereas differentiation into Th2 cells is promoted by IL-4, IL-5, IL-6, and IL-10. Furthermore, IL-4 secreted by Th2 cells acts on B cells and promotes the production of IgE, inducing the expression of IgE receptors in mast cells. Moreover, mast cells express cytokines, including IL-5 and GM-CSF, in response to IgE and stimulate eosinophils, which increase cytotoxicity and induce the secretion of chemical mediators [43, 44]. In contrast, IFN-*γ* and IL-2 secreted by Th1 cells have an antagonistic relationship with Th2 cell cytokines, such as IL-4, and inhibit IgE production by B cells [44]. The balance between Th1 and Th2 cell cytokines plays a role in maintaining normal body homeostasis (Figure 8).

In this study, the production of cytokines secreted by Th2 cells (IL-1*β*, IL-4, IL-5, IL-6, IL-10, and IL-13) and Th17 cells (IL17A, IL-17E, and IL-17F) significantly decreased, whereas the production of cytokines secreted by Th1 cells (IL-2 and IFN-*γ*) significantly increased in the serum and BALF of the CS73 group. The 7 : 3 ratio of chrysanthemum and skullcap extracts regulated the immune balance and significantly decreased the production of IgE, histamine, and TSLP, indicating the inhibitory effect on airway hyperresponsiveness.

Chrysanthemum extract blocked lipopolysaccharide- (LPS-) induced acute lung injury in mice, as demonstrated by the reduction in the number of WBCs, lymphocytes, and neutrophils [5]. Chrysanthemum contains several phytochemicals, including luteolin-7-glucoside, apigenin, and quercetin [8]. Luteolin-7-glucoside showed antiasthmatic activity in OVA-treated mice by downregulating Th2 cell cytokines and reducing prostaglandin *E*_2_ (PGE_2_) production [12]. Quercetin also had antiasthmatic activity, as demonstrated by decreased airway resistance and production of leukocytes, histamine, and phospholipase A2 in BALF of OVA-exposed guinea pigs [45]. Apigenin reduced OVA-increased IL-6, TNF-*α*, and IL-17A in the lungs and inhibited OVA-induced eosinophilia [46]. In addition to the protective effect of chrysanthemum on the lung, skullcap extracts also have a protective effect on the lungs. Skullcap extracts alleviated LPS-induced acute lung injury by reducing the production of nitric oxide (NO) and inflammatory cytokines and the ratio of lung wet/dry weight [6]. Skullcap extracts also include a variety of phytochemicals, such as baicalein and baicalin [9, 47]. Baicalein protected the lungs from myocardial ischemia and reperfusion by decreasing the levels of IL-1*β*, IL-6, and tumor necrosis factor- (TNF-) *α* [13]. Further, baicalin ameliorated avian pathogenic *Escherichia coli*-induced acute lung injury in chickens by deactivating nuclear factor kappa B (NF-*κ*B) [48]. Therefore, the protective effect of a mixture of chrysanthemum and skullcap extracts on the lung may be due to the production of phytochemicals with an anti-inflammatory effect and block the symptoms of lung-related diseases.

One major mechanism to induce asthma in an OVA-treated mouse model is NF-*κ*B activation-dependent inflammation. A previous study reported that when OVA was administered, NF-*κ*B *p*65 factors were translocated into the nucleus from the cytosol to transcribe inflammatory cytokines. Additionally, when OVA was administered, NF-*κ*B *p*65 factors were translocated into the nucleus from the cytosol to transcribe inflammatory cytokines [49]. Chrysanthemum extract not only decreased NF-*κ*B activity and the expression of inflammatory cytokines, such as TNF-*α*, IL-6, and inducible nitric oxide synthase (iNOS), but also blocked macrophage infiltration in obesity-induced inflammation in obese rats [50]. Skullcap extracts also suppressed inflammatory responses by blocking the translocation of NF-*κ*B in an LPS-induced acute lung injury mouse model [6]. Mitogen-activated protein kinase (MAPK) signaling is another mechanism related to asthma. OVA treatment stimulated the phosphorylation of extracellular signal-regulated kinase (ERK) and *p*38 MAPK proteins in BALB/c mice [49]. Chrysanthemum reduced p-ERK, p-*p*38, and p-c-Jun N-terminal kinase (JNK) levels in receptor activator of nuclear factor kappa-Β ligand- (RANKL-) treated osteoclasts [51]. In an acute lung injury model, skullcap extract inhibits MAPK protein phosphorylation [6]. In particular, a mixture of chrysanthemum and skullcap extracts significantly reduced the phosphorylation of JNK, *p*38, and ERK in LPS-treated RAW264.7 cells [7]. In this study, we investigated whether mixtures of chrysanthemum and skullcaps reduced the production of inflammatory cytokines in a mouse model, and the regulation of NF-*κ*B activity and the association with MAPK remain to be elucidated.

## 4. Conclusions

In conclusion, our study showed that a mixture of chrysanthemum and skullcap extracts can reduce inflammatory cytokine production in the serum and BALF of a mouse model of OVA-induced asthma. Furthermore, it can significantly reduce IgE, histamine, and TSLP production in a mouse model of asthma. Notably, chrysanthemum and skullcap extracts mixed at a 7 : 3 ratio were more effective than the other ratios. These extracts may be further developed as natural therapeutic agents for the treatment of asthma and improvement of bronchial health.

## Figures and Tables

**Figure 1:** HPLC chromatograms and UV spectrum of (a) luteolin 7-glucoside, (b) chrysanthemum extract, (c) baicalein, and (d) skullcap extract.

**Figure 2:** HPLC chromatograms and UV spectrum of luteolin 7-glucoside in mixtures of chrysanthemum and skullcap extracts in (a) 6 : 4, (b) 7 : 3, and (c) 8 : 2 ratios. HPLC chromatograms and UV spectrum of baicalein in mixtures of chrysanthemum and skullcap extracts in (d) 6 : 4, (e) 7 : 3, and (f) 8 : 2 ratios.

**Figure 3:** Effect of the extract mixture on white blood cells in BALF and eosinophil counts in the blood of mice with ovalbumin- (OVA-) induced asthma. The data are shown as the mean ± S.D.(*n* = 8 mice per group). ^*∗∗*^*p* < 0.01 compared with control.

**Figure 4:** Effect of the extract mixture on Th2 cytokine level of mice with ovalbumin (OVA-) induced asthma. The data are shown as the mean ± SD (*n* = 8 mice per group). ^*∗*^*p* < 0.05, ^*∗∗*^*p* < 0.01, and ^*∗∗∗*^*p* < 0.001 compared with the control.

**Figure 5:** Effect of the extract mixture on IL-17A, IL-17E, and IL-17F levels of ovalbumin (OVA-) induced asthma mice. The data are shown as the mean ± SD (*n* = 8 mice per group). ^*∗*^*p* < 0.05, ^*∗∗*^*p* < 0.01, and ^*∗∗∗*^*p* < 0.001 compared with the control.

**Figure 6:** Effect of the extract mixture on the IL-2 and IFN-*γ* levels of ovalbumin- (OVA-) induced asthma mice. The data are shown as the mean ± SD (*n* = 8 mice per group). ^*∗*^*p* < 0.05, ^*∗∗*^*p* < 0.01, and ^*∗∗∗*^*p* < 0.001 compared with the control.

**Figure 7:** Effect of the extract mixture on ovalbumin- (OVA-) specific IgE, histamine, and TSLP levels of OVA-induced asthma mice. The data are shown as the mean ± SD (*n* = 8 mice per group). ^*∗*^*p* < 0.05, ^*∗∗*^*p* < 0.01, and ^*∗∗∗*^*p* < 0.001 compared with the control.

**Figure 8:** Immunological mechanism of asthma.

**Table 1:** Effect of different mixing ratios of chrysanthemum and skullcap on immune factors.

Factor		Group^a,b^								
		6 : 4			7 : 3			8 : 2		
		50	100	200	50	100	200	50	100	200
White blood	BALF	—	↓	↓↓	—	↓↓	↓↓	—	↓	↓↓
Eosinophil		↓	↓	↓↓	↓↓	↓↓	↓↓	↓↓	↓	↓↓
IL-1*β*	Serum	—	↓	↓↓	↓	↓↓	↓↓	—	↓	↓
	BALF	—	↓	↓↓	↓	↓↓	↓↓	—	↓	↓

IL-4	Serum	—	↓	↓	↓↓	↓↓↓	↓↓↓	↓	↓↓↓	↓↓↓
	BALF	—	↓	↓	↓↓	↓↓↓	↓↓↓	↓	↓↓↓	↓↓↓

IL-5	Serum	↓	↓	↓↓	↓↓	↓↓↓	↓↓↓	—	↓	↓↓↓
	BALF	↓	↓	↓↓	↓↓	↓↓↓	↓↓↓	—	↓	↓↓↓

IL-6	Serum	↓↓	↓↓	↓↓↓	↓↓	↓↓↓	↓↓↓	↓↓	↓↓↓	↓↓↓
	BALF	—	↓	↓↓	↓	↓↓	↓↓↓	—	↓	↓

IL-10	Serum	↓	↓↓	↓↓↓	↓↓	↓↓↓	↓↓↓	↓↓	↓↓↓	↓↓↓
	BALF	—	↓	↓↓	↓	↓↓	↓↓	↓	↓↓	↓↓↓

IL-13	Serum	—	↓↓	↓↓↓	↓	↓↓↓	↓↓↓	↓	↓↓	↓↓↓
	BALF	—	↓↓	↓↓↓	↓	↓↓↓	↓↓↓	↓	↓↓	↓↓↓

IL-17A	Serum	—	—	↓↓	↓	↓↓↓	↓↓↓	↓	↓↓	↓↓↓
	BALF	—	—	↓↓	↓	↓↓↓	↓↓↓	↓	↓↓	↓↓↓

IL-17F	Serum	—	↓	↓↓	↓	↓	↓↓	—	↓↓	↓↓
	BALF	—	↓↓	↓↓↓	↓↓	↓↓	↓↓↓	—	↓↓↓	↓↓↓

IL-17E	Serum	—	—	↓	↓↓	↓↓↓	↓↓↓	↓	↓↓	↓↓
	BALF	—	—	↓	↓↓	↓↓↓	↓↓↓	↓	↓↓	↓↓

IL-2	Serum	—	↑	—	—	↑	↑↑	—	—	—
	BALF	—	↑	—	—	↑	↑↑	—	—	—

IFN-*γ*	Serum	↑	↑↑	↑↑	↑	↑↑	↑↑↑	↑	↑	↑↑
	BALF	↑	↑↑	↑↑	↑	↑↑	↑↑↑	↑	↑	↑↑

IgE	Serum	—	—	↓↓	↓	↓	↓↓	↓	↓	—
	BALF	↓	↓	↓↓↓	↓↓	↓↓	↓↓↓	↓↓	↓↓	—

Histamine	Serum	—	↓	↓	↓	↓↓	↓↓	↓	—	—
	BALF	—	↓	↓	↓	↓	↓	↓	—	—

TSLP	Serum	↓↓	↓	↓	↓	↓↓	↓↓	—	—	↓
	BALF	↓↓	↓	↓	—	↓↓	↓↓	—	—	↓

BALF: bronchoalveolar lavage fluid; IL: interleukin; TSLP: thymic stromal lymphopoietin. ^a^The chrysanthemum and skullcap extracts were mixed in a 6 : 4, 7 : 3, or 8 : 2 ratio (row 2). ^b^The mice were orally administered 50, 100, or 200 mg/kg BW of the mixture (row 3).

## Data Availability

The data used to support the findings of this study are available from the corresponding author upon request.
